This article has been retracted.

# MicroRNA-130b promotes lung cancer progression via PPARγ/VEGF-A/BCL-2-mediated suppression of apoptosis

**DOI:** 10.1186/s13046-016-0382-3

**Published:** 2016-07-01

**Authors:** Jianwei Tian, Liping Hu, Xiao Li, Jian Geng, Meng Dai, Xiaoyan Bai

**Affiliations:** State Key Laboratory for Organ Failure Research, Division of Nephrology, Nanfang Hospital, Southern Medical University, Guangzhou, 510515 Guangdong China; Department of Emergency, Nanfang Hospital, Southern Medical University, Guangzhou, Guangdong China; Department of Pathology, Nanfang Hospital, Southern Medical University, Guangzhou, Guangdong China; Health Management Center, Nanfang Hospital, Southern Medical University, Guangzhou, Guangdong China

**Keywords:** MicroRNA-130b, PPARγ, BCL-2, Apoptosis, NSCLC

## Abstract

**Background:**

The prognosis of non-small-cell lung cancer (NSCLC) is poor yet mechanistic understanding and therapeutic options remain limited. We investigated the biological and clinical significance of microRNA-130b and its relationship with apoptosis in NSCLC.

**Methods:**

The level of microRNA-130b in relationship with the expression of PPARγ, VEGF-A, BCL-2 and apoptosis were analyzed in 91 lung cancer patient samples using immunohistochemistry and terminal deoxynucleotidyl transferase dUTP nick end labeling (TUNEL) assay on tissue microarrays. Gain and loss-of-function studies were performed to investigate the effects of microRNA-130b, peroxisome proliferator-activated receptor γ (PPARγ) or vascular endothelial growth factor-A (VEGF-A) on biological functions of lung cancer cells using in vitro and in vivo approaches.

**Results:**

MicroRNA-130b up-regulation conferred unfavorable prognosis of lung cancer patients. Notably, microRNA-130b targeted PPARγ and inhibiting microRNA-130b markedly repressed proliferation, invasion and metastasis of lung cancer cells, leading to increased apoptosis. MicroRNA-130b-dependent biologic effects were due to suppression of PPARγ that in turn activated BCL-2, the key mediator of anti-apoptosis. Administration of microRNA-130b mimic to mouse xenografts promoted tumor growth. In vitro and in vivo, miR-130b enrichment associated with down-regulation of PPARγ, up-regulation of VEGF-A and BCL-2, and decreased apoptosis.

**Conclusions:**

The present study demonstrates that microRNA-130b promotes lung cancer progression via PPARγ/VEGF-A/BCL-2-mediated suppression of apoptosis. Targeting microRNA-130b might have remarkable therapeutic potential for lung cancer therapy.

**Electronic supplementary material:**

The online version of this article (doi:10.1186/s13046-016-0382-3) contains supplementary material, which is available to authorized users.

## Background

Several microRNAs (miRNAs), such as miR-21, miR-152, miR-148b and miR-208a, play critical roles in lung cancer progression through modulating growth, apoptosis, metastasis and invasion [1–4]. A recent study has identified microRNA-130 (miR-130) as a contributor in mesenchymal differentiation, hypoxic response modulation and tumorigenesis in colorectal cancer [5]. MiR-130b has also been documented in several other kinds of tumors, with up-regulation in melanoma [6], but down-regulation in endometrial cancer [7] and pituitary adenomas [8].

Peroxisome proliferator-activated receptor γ (PPARγ), acting as a tumor suppressor, exerts an essential role in modulating tumor proliferation, differentiation, apoptosis and invasion [9–11]. Combined treatment with the cyclo-oxygenase-2 (Cox-2) inhibitor niflumic acid and PPARγ ligand ciglitazone induces endoplasmic reticulum stress/caspase-8-mediated apoptosis in human lung cancer cells [12]. Treatment of human NSCLC lines with PPARγ ligands results in growth arrest, loss of capacity and induction of apoptosis [13]. Additionally, PPAR-response element (PPRE) has been identified in the human vascular endothelial growth factor-A (VEGF-A) promoter region [14] and PPARγ ligands have been documented to down-regulate VEGF-A expression in prostate cancer [15]. VEGF-A up-regulation has been implicated in lung carcinogenesis [16] and correlates with apoptosis by driving the expression of BAX [17]. However whether VEGF-A interacts with BCL-2, a classical anti-apoptotic gene, in modulating lung cancer cell apoptosis remains unclear.

Studies have revealed that miR-130b promotes tumor aggressiveness by suppressing PPARγ but promotes VEGF-A expression and epithelial to mesenchymal transition (EMT) in hepatocellular [18] and colorectal cancer [5]. In terms of the correlations between PPARγ, VEGF-A and apoptosis, we hypothesize that miR-130b suppresses PPARγ and promotes lung cancer progression via VEGF-A/BCL-2-mediated inhibition of apoptosis. We also investigated the correlation between miR-130b expression and lung cancer patient’s prognosis and survival. Mechanisms of miR-130b/PPARγ-mediated apoptosis and lung cancer progression were also explored.

## Methods

### Patients and specimens

Total 91 NSCLC patients undergoing treatment in Nanfang Hospital in Guangzhou China from 2012 to 2015 were selected. This study was specifically approved by the Southern Medical University Ethnics Committee. Informed consent was obtained from all individual participants included in the study. The overall survival time after tumor resection was 57.9 months (range 19–98 months). Specimens from these patients were obtained from the Department of Pathology and the Department of Thoracic Surgery in Nanfang Hospital. Thirty-six snap frozen fresh tumor samples and matched normal lung tissues (10 cm from the tumor) obtained from among the 91 specimens were also available for the study. Clinical pathologic characteristics of the patients were based on the World Health Organization criteria [19], as was described in Table 1.

**Table 1:** Clinicopathologic characteristics of patients with lung cancer

Characteristics		All patients (*N* = 91) (%)
Gender		
	Male	38(42 %)
	Female	53(58 %)
Smoking Status		
	Nonsmoker	19(21 %)
	Smoker	72(79 %)
Tumor Location		
	Central	37(41 %)
	Peripheral	54(59 %)
Tumor Subtypes		
	Adenocarcinoma	51(56 %)
	Squamous Cell Carcinoma	40(44 %)
Differentiation		
	High	47(52 %)
	Moderate-Poor	44(48 %)
LN Metastasis		
	Yes	55(60 %)
	No	36(40 %)
Tumor Size		
	>3 cm	57(63 %)
	<3 cm	34(37 %)
TNM Stage		
	I-II	39(43 %)
	III-IV	52(57 %)
Mean Survival Time (months)		57.96

Total RNA from tissues of lung cancer patients and healthy controls was extracted using Trizol Reagent (Invitrogen, Carlsbad, CA). The synthetic oligonucleotide (3’-UUUCAUGUCGAUUUCAUUUCAUG-5’) non-existent in humans was spiked-in for quality control before miRNAs extraction according to the manufacturer’s instructions. The thermal cycle (Ct) values for a serial dilution of these miRNAs were assessed. All experiments were repeated in triplicate.

### Immunolabeling

Tissue microarray construction, immunohistochemical staining and immunofluorescence co-labeling were carried out according to previously published procedures [20]. Briefly, samples were stained with the antibodies to PPARγ, VEGF-A and BCL-2 (Abcam, Cambridge) followed by EnVision/HRP Kit (Dako, Carpinteria, CA) and imaged with a BX51 light microscope (Olympus, Tokyo). The staining intensity was scored according to previously procedures [21].

### Cell culture studies

A549 (adenocarcinoma) and H520 (squamous cell carcinoma) lung cancer cells were obtained from American Type Culture Collection (ATCC, Manassas, VA) and maintained in RPMI 1640 supplemented with 1 % penicillin/streptomycin and 10 % fetal bovine serum (FBS) in 5 % CO_2,_ 37°C cell culture incubator.

### Transfection of miRNA inhibitor and small interfering RNA

MiR-130b inhibitor (anti-M), miR-130b mimic, or the appropriate negative controls of miRNA inhibitor (anti-MC) and miRNA mimic were purchased from GenePharma (Shanghai, China). Anti-M and anti-MC were transfected at a final concentration of 50–100 nM in the cells using HiPerFect Transfection Reagent (Qiagen, Hilden, Germany) according to the manufacturer’s recommendations. Expression of PPARγ and VEGF-A were knocked down with small interfering RNA (siRNA) duplexes using Oligofectamine (Invitrogen, Carlsbad, CA). The target sequences for PPARγ and VEGF-A mRNA were shown in Table 2. Non-targeting siRNA pool (D-001206-13-05; Dharmacon, Fisher Scientific, Pittsburgh, PA) was used as a negative control. Cells were harvested 72 hours post transfection for analysis.

**Table 2:** Target sequences for *PPARγ* and *VEGF-A* mRNA

Genes	Target sequences
*PPARγ*	5’-AAUAUGACCUGAAGCUCCAAGAAUAAG-3’
*VEGF-A*	5’-TGCTGTGAAGATGTACTCTATCTCGTGTTTTGGCCACTGACTGACACGAGATAGTACATCTTCA-3’

### Luciferase reporter assay

The predicted 3'-untranslated region (UTR) sequence of *PPARγ* and *BCL-2* interacting with miR-130b and *VEGF-A*, respectively, and mutated sequences within the predicted target sites were synthesized and inserted into the pRL-TK control vector (Promega, Madison, WI). H520 cells transfected with 120 ng anti-miR-130b, *VEGF-A* siRNA or negative controls, followed by co-transfection with 30 ng of the wild-type or mutant 3'-UTR of the mRNA of *PPARγ* or *BCL-2* using 0.45 μL of Fugene (Promega, Madison, WI). Luciferase assay was carried out using Dual-Luciferase Assay System (Promega, Madison, WI). Data were normalized by the ratio of firefly and Renilla luciferase activities measured at 48 h post-transfection.

### Drug treatment

VEGF-A inhibitor (bevacizumab, 2.5 μM) and PPARγ inhibitor, GW9662 (20 μM, Sigma-Aldrich, St. Louis, MO) were used to treat A549 and H520 cells for 72 h and harvested for further analysis.

### Cell proliferation assay

Cell proliferation analysis was performed in triplicate using a CellTiter 96 Non-Radioactive Cell Proliferation Assay Kit (Promega, Madison, WI) following the manufacturer’s protocols.

### Cell migration assay

Cells (1.0 × 10^6^ cells/ml) in serum-free medium were added to the top chamber of 24-well transwell plates (8 mm pore size; Corning Star, Cambridge, MA) and 600 μl of complete medium with 10 % FBS into the bottom chamber. The assembled chamber was incubated at 37 °C in a humidified, 5 % CO_2_ cell culture incubator for 24 h, fixed with 10 % formalin and stained with hematoxylin and eosin staining for visualization.

### Cell invasion assay

Cells (5.0 × 10^4^ cells/mL) were plated in 6-well plates and grown to over 90 % confluence. The monolayer of cells was scratched with a 200 μL pipette tip to create a wound gap, and treated with miR-130b inhibitor, siRNAs of *PPARγ* or *VEGF-A*, and control (0.1 % DMSO) at indicated time points. The same visual field was photographed using BX41 light microscope (10× objective) throughout the experiment. Wound closure was calculated as follows: Wound closure (%) = Gap (T-T0)/GapT0 × 100 % (where T is the treatment time and T0 is the time that the wound was induced).

### In vitro plate-colony formation assay

Cells (200 cells/well) were plated in a six-well tissue culture plate and cultured for two weeks. Colonies with ≥50 cells were counted and plate colony formation efficiency was evaluated according to the following formula: (number of colonies/number of cells inoculated) × 100 %. Triplicate samples from each group of cells were examined and colonies were counted by two individuals (XL and JG).

### Apoptosis assay and cell cycle analysis using flow cytometry

Fixed cells were stained with the Annexin V-PE/7-AAD apoptosis kit (559763, BD Biosciences, Franklin Lakes, NJ) and apoptosis was evaluated by examining the percentage of apoptotic cells. Data acquisition and analysis were performed using Cell Quest software via a FACScan flow cytometer (BD Biosciences, Franklin Lakes, NJ). The results were analyzed with the ModFit 3.0 software (Verity Software House, Topsham, ME). All experiments were repeated in triplicate.

### TUNEL assay

Cells subjected to siRNA transfection or untreated cells were fixed with 4 % paraformaldehyde and detected using terminal deoxynucleotidyl transferase dUTP nick end labeling (TUNEL) assay with an Apoptag Peroxidase in Situ Apoptosis Detection kit (Chemicon International, Temecula, CA) as described previously [22].

### qRT-PCR analysis

qRT-PCR analysis was carried in triplicate with Power PCR SYBR Green Master Mix (Applied Biosystems, Carlsbad, CA) using the ABI PRISM 7500 FAST Real-TIME PCR System (Applied Biosystems, Carlsbad, CA) with results normalized to U6 or β-actin expression. The relative expression was calculated using the ΔΔC_T_ method. Primer sequences used in qRT-PCR were listed in Table 3.

**Table 3:** Primer sets used in real time RT-PCR

Genes	Forward primer	Reverse primer
*PPARγ*	5'-AGGTAAGGAGTCAGAAACGGG-3'	5'-TCGTTAAAGGCTGACTCTCGT-3'
*VEGF-A*	5'-TCACCAAGGCCAGCACATAG-3'	5'-GAGGCTCCAGGGCATTAGA-3'
*BCL-2*	5'-CATGTGTGTGGAGAGCGTCA-3'	5'-GAAATCAAACAGAGGCCGCA-3'
β-ACTIN	5'-ATGATGATATCGCCGCGCTC-3'	5'-TCGATGGGGTACTTCAGGGT-3'

The specific miR-130b miScript Primer Assays (Qiagen, Hilden, Germany) were used for miRNA expression analysis. RNA was reverse transcribed using miRScript PCR System and analyzed by qRT-PCR with the miScript SYBR Green PCR Kit. MiR-130b levels were calculated as fold change (2^-ΔΔCT^) with respect to normal controls. The mean value of miR-130b expression in tumor tissues was calibrated to the levels detected in normal control tissues. Target-specific reverse transcription and Taqman microRNA assays were performed using the Hairpin-itTM miRNA qPCR Quantitation Kit (GenePharma, Suzhou) according to the protocol. The reactions were performed using the ABI PRISM 7500 FAST Real-TIME PCR System (Applied Biosystems, Carlsbad, CA). The relative expression of miR-130b was shown as fold difference relative to U6. The average value between 0.5 to 1.0 was regarded as miR-130b low and the value between 1.0 to 1.6 as miR-130b high. The 2^-ΔΔCt^ method was used to calculate the relative expression. All experiments were performed in triplicate.

### Western blot analysis and immunoprecipitation

Cell lysates from each experimental group were separated in parallel on two 10 % denaturing SDS-PAGE gels, transferred onto nitrocellulose membranes, blocked with 5 % non-fat milk in 0.1 % tris buffered saline with Tween-20 (TBST), and probed with antibodies to PPARγ, VEGF-A, and BCL-2, followed by incubation with appropriate secondary antibodies. The probed membrane was exposed and protein bands were visualized on X-ray films (Kodak X-OMAT BT, Rochester, NY). Immunoprecipitation was performed as previously described [23].

### In Vivo Studies of Tumorigenicity

Male balb/c nude mice were kept in the Animal Center of Nanfang Hospital, Guangzhou, China according to the policies of the Committee for Animal Usage. To evaluate in vivo tumor growth, A549 cells with miR-130b mimic or appropriate controls (2 ng/mm^3^) were injected subcutaneously into the left flanks of ten mice. Thirty days after the injection, mice were euthanized and tumor growth was evaluated. Tumor volume (mm^3^) was calculated as (W2 × L)/2. Immunohistochemical staining for PPARγ, VEGF-A and BCL-2 were performed on mouse tissue specimens according to the previously mentioned method [21].

### Statistical analysis

Data are expressed as mean ± standard deviation (SD) values. Correlations between expressions of miR-130b and PPARγ, VEGF-A and BCL-2 and lung cancer patients’ clinical pathological characteristics were analyzed using two-sided Fisher’s Exact Test. Pearson Correlation Analysis and Independent-Samples T Test were used to evaluate the correlation and significance between the expression of VEGF-A and PPARγ or BCL-2. Overall patient survival was calculated from the time of surgery to the time of death or to the time of last follow-up, at which point the data were censored. Kaplan-Meier method and the log-rank test were used to evaluate the difference between high and low miR-130b expression subgroups and the overall survival curves were generated. SPSS 13.0 (SPSS Inc., Chicago, IL) was used for all statistical analysis. A *p* < 0.05 was regarded as statistically significant.

## Results

### High miR-130b expression confers unfavorable prognosis of lung cancer patients

To investigate whether miR-130b expression predicts patients’ prognosis, we examined miR-130b expression in tissues of lung cancer patients. We found increased miR-130b expression in lung cancer tissues compared with corresponding normal lungs. By qRT-PCR (Fig. 1a), low level of miR-130b was detected in 46 cases and high miR-130b expression was found in 45 cases. In lung cancer tissues, high miR-130b level corresponded with low PPARγ, high VEGF-A and BCL-2, and decreased apoptosis (Figs. 1b, c and d). Kaplan-Meier survival analysis demonstrated that patients with high miR-130b expression had a shorter overall survival time compared to patients with low miR-130b expression (Fig. 1e, 48.4 vs. 67.8 months, *p* < 0.001). Immunofluorescence co-labeling and Pearson correlation analysis (Fig. 2) revealed that PPARγ expression negatively correlated with VEGF-A (*r* = −0.351, *p* = 0.001), and VEGF-A positively correlated with BCL-2 (*r* = 0.328, *p* = 0.002). MiR-130b expression associated with differentiation (*p* = 0.002) and TNM stage (*p* = 0.025) of lung cancer patients (Table 4).

**Table 4:** Correlation between MiR-130b and patient clinicopathological characteristics

Items		MiR-130b (*N* = 91)		*p*
		Low (*N* = 46)	High (*N* = 45)	
Gender				0.929
	Male	19	19	
	Female	27	26	
Smoking Status				0.303
	Nonsmoker	12	7	
	Smoker	34	38	
Tumor Location				0.327
	Central	21	16	
	Peripheral	25	29	
Differentiation				0.002
	High	31	16	
	Moderate-Poor	15	29	
LN Metastasis				0.026
	Yes	33	22	
	No	13	23	
Tumor Size				0.002
	>3 cm	36	21	
	<3 cm	10	24	
TNM Stage				0.025
	I-II	25	14	
	III-IV	21	31	

*p* values listed are derived from χ^2^ test

These results suggested that miR-130b could be used as a marker to predict lung cancer patients’ prognosis.

**Fig. 1:** High miR-130b expression confers unfavorable prognosis of lung cancer patients. **a** MiR-130b expression in lung cancer tissues. **b** MiR-130b expression in relation to the expression of PPARγ, VEGF-A and BCL-2. **c** Representative TMA sections stained for PPARγ, VEGF-A and BCL-2 by immunohistochemistry (scale bar, 100 μm), and apoptosis by TUNEL assay (scale bar, 50 μm). **d** Correlations between miR-130b level and PPARγ, VEGF-A, BCL-2 or apoptosis. **e** A shorter overall survival time in patients with high miR-130b. NL, normal lung; AD, adenocarcinoma; SQ, squamous cell carcinoma; TUNEL, terminal deoxynucleotidyl transferase-mediated uridine 5’-triphosphate-biotin nick end labeling. *p < 0.05, #*p* < 0.001

**Fig. 2:** The expression of VEGF-A in correlation with PPARγ and BCL-2. **a** Representative sections co-labeled for PPARγ (green) and VEGF-A (red) and **b** the quantification analysis. **c** Negative correlation between PPARγ and VEGF-A expression. **d** Representative sections co-labeled for VEGF-A (red) and BCL-2 (green) and **e** the quantification analysis. **f** Positive correlation between VEGF-A and BCL-2. Scale bar, 50 μm. Each bar represents the mean ± SD. Results are representative of three independent experiments. *p < 0.05, #*p* < 0.001

### MiR-130b inhibition attenuates lung cancer cell aggressiveness via PPARγ/VEGF-A/BCL-2-mediated enhancement of apoptosis

To decipher whether miR-130b promotes lung cancer progression and underlying mechanisms, we examined the effect of miR-130b inhibitor on the biological features of lung cancer cells and relationships with apoptosis. Inhibition of miR-130b increased PPARγ expression but decreased VEGF-A and BCL-2 as confirmed by immunofluorescence microscopy (Fig. 3a and b). Compared with negative controls, anti-miR-130b caused 23.7 % increase in the mRNA level of *PPARγ*, but 47.3 % and 43.2 % reduction in *VEGF-A* and *BCL-2* as detected by qRT-PCR (Fig. 3c). Western blot analysis demonstrated that anti-miR-130b increased the level of PPARγ by 65.2 % but decreased VEGF-A and BCL-2 by 60.8 % and 38.5 %, respectively (Fig. 3d). To further demonstrate that miR-130b targeted PPARγ in lung cancer cells, we investigated whether miR-130b interacted with the 3’-UTR of PPARγ mRNA using a dual-luciferase reporter assay. As shown, miR-130b depletion led to a significant increase in the luciferase activity of the wild-type reporter but not the mutant (Fig. 3e). A significantly slower proliferation rate was observed in lung cancer cells treated with anti-miR-130b compared with controls (Fig. 3f). MiR-130b depletion inhibited the ability of cells to invade (Fig. 3g), migrate (Fig. 3h) and form colonies (Fig. 3i). Anti-miR-130b caused 1.48-fold increase in the number of apoptotic cells compared with control cells by flow cytometric analysis (Fig. 3j). TUNEL assay revealed that miR-130b abrogation significantly enhanced apoptosis and caused 52.6 % increase in the apoptotic rate (Fig. 3k). Conversely, miR-130b mimic had the opposite effects (Additional file 1: Supplementary Figure). These results collectively suggested that miR-130b inhibition decreased lung cancer cell aggressiveness via PPARγ/VEGF-A/BCL-2-mediated enhancement of apoptosis.

**Fig. 3:** MiR-130b inhibition attenuates lung cancer cell aggressiveness via PPARγ/VEGF-A/BCL-2-mediated enhancement of apoptosis. **a** Representative images of A549 cells treated with anti-miR-130b and co-labeled for PPARγ (green) and VEGF-A (red) (scale bar, 50 μm). **b** Representative images of A549 cells treated with anti-miR-130b and labeled for BCL-2 (green) (scale bar, 50 μm). **c** and **d** Anti-miR-130b increased PPARγ, but decreased VEGF-A and BCL-2. **e** MiR-130b and its putative binding sequence in the PPARγ 3'-UTR. The mutant PPARγ binding site was generated in the complementary site for the seed region of miR-130b. Anti-miR-130b caused a significant increase in the luciferase activity of wt 3'-UTR of *PPARγ*. **f** A slower proliferation rate in cells treated with anti-miR-130b compared with controls. **g** Decreased number of invaded cells with anti-miR-130b treatment (scale bar, 100 μm). **h** Shorter migrated distance in cells treated with anti-miR-130b at indicated time points. **i** Decreased colonies in cells treated with anti-miR-130b at 48 hours time point. **j** Increased apoptotic cells treated with anti-miR-130b compared with controls. **k** Increased apoptotic rate in cells treated with anti-miR-130b (scale bar, 50 μm). Anti-MC: anti-miR-130b control; anti-M: anti-miR-130b; TUNEL, terminal deoxynucleotidyl transferase-mediated uridine 5’-triphosphate-biotin nick end labeling; UTR, untranslated region; wt, wild type; mt, mutant type. Each bar represents the mean ± SD. Results are representative of three independent experiments. *p < 0.05, #*p* < 0.001

### *PPARγ* silencing enhances lung cancer cell aggressiveness via VEGF-A/BCL-2-mediated suppression of apoptosis

Next we knocked down *PPARγ* in lung cancer cells to investigate whether *PPARγ* mediated apoptosis through the VEGF-A/BCL-2 pathway and whether PPARγ had feedback regulation of miR-130b expression. We found that *PPARγ* silencing increased the expression of VEGF-A and BCL-2 as demonstrated by immunofluorescence microscopy (Fig. 4a and b). Compared with negative controls, *PPARγ* siRNAs (#1 and #2) decreased the mRNA level of *PPARγ* (46.1 and 39.5 %), but increased *VEGF-A* (23.8 and 21.3 %) and *BCL-2* (12.1 and 11.3 %), respectively, as shown by qRT-PCR (Fig. 4c). *PPARγ* siRNAs (#1 and #2) decreased the protein level of *PPARγ* (87.4 and 89.8 %), but increased *VEGF-A* (89.9 and 88.7 %) and *BCL-2* (86.8 and 85.9 %), respectively, as detected by Western blot analysis (Fig. 4d). A significantly faster proliferation rate and more Ki-67 positive cells were observed in *PPARγ*-silenced cells as compared with control cells (Fig. 4e and f). *PPARγ* silencing promoted the invasion (Fig. 4g) and migration ability (Fig. 4h) of lung cancer cells with increased ability to form colonies (Fig. 4i). *PPARγ* siRNAs caused significant decrease in the number of apoptotic cells (8.8 and 8.6 %) compared with control cells (11.9 %) by flow cytometric analysis (Fig. 4j). *PPARγ* silencing caused 58.3 and 54.7 % decrease in the cell apoptotic rate by TUNEL assay (Fig. 4k). However, *PPARγ* siRNAs had no effects on the expression level of miR-130b (Fig. 4l). These results suggested that *PPARγ* depletion promoted the aggressiveness of lung cancer cells through VEGF-A/BCL-2-mediated suppression of apoptosis. However, PPARγ did not have feedback regulation on miR-130b.

**Fig. 4:** *PPARγ* silencing enhances lung cancer cell aggressiveness via VEGF-A/BCL-2-mediated suppression of apoptosis. **a** Representative images of A549 cells treated with *PPARγ* siRNAs and co-stained for PPARγ (green) and VEGF-A (red) (scale bar, 50 μm). **b** Representative images of A549 cells treated with *PPARγ* siRNAs and stained for BCL-2 (green) (scale bar, 50 μm). **c** and **d** *PPARγ* siRNAs (#1 and #2) decreased PPARγ, but increased *VEGF-A* and *BCL-2*, respectively. **e** A faster proliferation rate in *PPARγ*-silenced cells compared with controls. **f** More Ki-67 positive proliferative cells (green) in *PPARγ*-silenced cells (scale bar, 100 μm). **g** Increased number of invaded *PPARγ*-silenced cells compared with controls (scale bar, 100 μm). **h** Longer migrated distance in *PPARγ*-silenced cells at indicated time points. **i** Increased colonies in *PPARγ*-silenced cells at 48 hours time point. **j** Decreased apoptotic cells (8.8 and 8.6 %) compared with controls (11.9 %). **k** Decreased apoptotic rate in *PPARγ*-silenced cells (scale bar, 100 μm). **l** No effect of *PPARγ* siRNAs on the level of miR-130b. NT siRNA: non-targeting small interference RNA; TUNEL, terminal deoxynucleotidyl transferase-mediated uridine 5’-triphosphate-biotin nick end labeling. Each bar represents the mean ± SD. Results are representative of three independent experiments. *p < 0.05, #*p* < 0.001

### Knockdown of *VEGF-A* reduces lung cancer cell aggressiveness via *BCL-2*-mediated activation of apoptosis in vitro

To further investigate whether *VEGF-A* induced cell apoptosis via *BCL-2* inhibition, *VEGF-A* siRNAs were used to knock down the expression of VEGF-A. Downstream gene expressions and biological features of cells were examined. Immunofluorescence microscopy revealed that *VEGF-A* siRNAs decreased the expression of BCL-2 and the two molecules co-localized with each other (arrowheads) (Fig. 5a). Compared with negative control cells, *VEGF-A* siRNAs (#1 and #2) decreased the mRNA level of *VEGF-A* (28.3 and 29.2 %) and *BCL-2* (65.6 and 63.3 %), respectively, by qRT-PCR (Fig. 5b). *VEGF-A* siRNAs (#1 and #2) decreased the protein level of VEGF-A (63.8 and 91.4 %) and BCL-2 (88.1 and 60.8 %), respectively, by Western blot analysis (Fig. 5c). *VEGF-A* siRNA led to a significant decrease in the luciferase activity of wt 3'-UTR of *BCL-2* (Fig. 5d). Furthermore, *VEGF-A* siRNAs slowed cell growth (Fig. 5e and f), reduced the ability of cells to migrate (Fig. 5g), invade (Fig. 5h) and form colonies (Fig. 5i). *VEGF-A* siRNAs caused significant increase in the number of apoptotic cells (17.0 and 17.3 %) as detected by flow cytometric analysis (Fig. 5j) and 30.5 and 28.1 % increase in the apoptotic rate by TUNEL assay (Fig. 5k). However, *VEGF-A* siRNAs had no effects on miR-130b expression (Fig. 5l). These results demonstrated that VEGF-A silencing induced cell apoptosis via inhibition of BCL-2. However, VEGF-A had no feedback regulation on miR-130b in lung cancer cells.

**Fig. 5:** Knockdown of *VEGF-A* reduces lung cancer cell aggressiveness via *BCL-2*-mediated activation of apoptosis in vitro. **a** Representative images stained for VEGF-A (red) and BCL-2 (green) and co-localization (yellow, arrowheads) (scale bar, 50 μm). **b** and **c** *VEGF-A* siRNAs (#1 or 2) decreased *VEGF-A* and *BCL-2*, respectively. **d** *VEGF-A* siRNAs caused a significant decrease in the luciferase activity of wt 3'-UTR of *BCL-2*. **e** A slower proliferation rate in cells treated with *VEGF-A* siRNAs compared with controls. **f** Fewer Ki-67 positive cells in *VEGF-A* silenced cells compared with controls (scale bar, 100 μm). (**g**) Decreased number of invaded cells with *VEGF-A* siRNAs (scale bar, 100 μm). (**h**) Shorter migrated distance in cells treated with *VEGF-A* siRNAs at indicated time points. (**i**) Decreased colonies in *VEGF-A* silenced cells at 48 hours time point. **j** Increased apoptotic cells (17.0 and 17.3 %) compared with controls (11.9 %). **k** Increased apoptotic rate in *VEGF-A* silenced cells (scale bar, 50 μm). **l** No effect of *VEGF-A* siRNAs on the level of miR-130b. NT siRNA: non-targeting small interference RNA. Each bar represents the mean ± SD. Results are representative of three independent experiments. *p < 0.05, #*p* < 0.001

### PPARγ antagonism abolishes the effect of miR-130b inhibition on VEGF-A/BCL-2-mediated apoptosis

To further explore whether miR-130b targets PPARγ in mediating apoptosis, we treated lung cancer cells with PPARγ antagonist GW9662 and examined the downstream effects. Western blot analysis demonstrated that anti-miR-130b up-regulated the expression level of PPARγ but down-regulated VEGF-A and BCL-2. GW9662 abolished the effect of miR-130b inhibition on the expression of VEGF-A and BCL-2 (Fig. 6a). Treatment with VEGF-A inhibitor bevacizumab (2.5 μM) down-regulated the expression of BCL-2 in a time- (Fig. 6b) and dose-dependent manner (Fig. 6c). Immunoprecipitation analysis revealed that bevacizumab significantly inhibited the interaction between PPARγ and VEGF-A upon miR-130b inhibition (Fig. 6d), suggesting VEGF-A acted as the downstream of PPARγ in mediating the cascade of events. Further studies also demonstrated that VEGF-A interacted with BCL-2 upon PPARγ inhibition (Fig. 6e). Flow cytometric analysis (Fig. 6f, upper panels) and the TUNEL assay (Fig. 6f, middle panels) demonstrated that PPARγ antagonist GW9662 attenuated the effect of miR-130b inhibition on VEGF-A/BCL-2-mediated apoptosis (Fig. 6f, lower panels). Taken together, these results suggested that PPARγ functioned as a critical regulator in miR-130b mediated lung cancer apoptosis through the VEGF-A/BCL-2 pathway.

**Fig. 6:** PPARγ antagonism dampens the effect of miR-130b inhibition on VEGF-A/BCL-2-mediated apoptosis. **a** Requirement of PPARγ in miR-130b mediated expressions of VEGF-A and BCL-2. **b** Bevacizumab down-regulated BCL-2 in a time- and **c** dose-dependent manner. **d** Interaction between PPARγ and VEGF-A by immunoprecipitation. **e** Interaction between VEGF-A and BCL-2 by immunoprecipitation. **f** Apoptosis was increased by anti-miR-130b but decreased by GW9662. Attenuation of the effect of miR-130b inhibition on apoptosis by GW9662. Scale bar, 100 μm. Anti-M: anti-miR-130b; bev.: bevacizumab; TUNEL, terminal deoxynucleotidyl transferase-mediated uridine 5’-triphosphate-biotin nick end labeling. Each bar represents the mean ± SD. Results are representative of three independent experiments. *p < 0.05, #*p* < 0.001

### MiR-130b promotes tumor growth and suppresses apoptosis via PPARγ/VEGF-A/BCL-2 signaling in mouse xenografts

To investigate the effect of miR-130b on tumor growth in vivo, miR-130b mimic or controls was injected subcutaneously into the mouse. We found that miR-130b mimic significantly increased the tumor volume of A549 mouse xenografts compared with controls in one month time (Fig. 7a and b). MiR-130b mimic decreased the protein level of PPARγ by 51.7 %, but increased VEGF-A and BCL-2 by 41.3 and 52.6 %, respectively, confirmed by immunohistochemistry (Fig. 7c) and quantification of the staining intensity (Fig. 7d). MiR-130b mimic reduced the apoptotic rate by 52.6 % (Fig. 7e), decreased PPARγ mRNA level by 53.3 %, increased VEGF-A and BCL-2 by 62.8 and 49.3 %, respectively, as detected by qRT-PCR (Fig. 7f). MiR-130b mimic decreased PPARγ protein level by 87.2 %, but increased VEGF-A and BCL-2 by 96.4 and 90.1 %, respectively, by Western blot analysis (Fig. 7g). These data confirmed the in vitro findings and further supported the notion that miR-130b promoted tumor growth and suppressed apoptosis via PPARγ/VEGF-A/BCL-2 signaling.

**Fig. 7:** MiR-130b promotes tumor growth and suppresses apoptosis via PPARγ/VEGF-A/BCL-2 signaling in A549 mouse xenograft. **a** and **b** Larger tumor volume treated with miR-130b mimic compared with the control at day 30. **c** MiR-130b mimic decreased PPARγ and apoptosis, but increased VEGF-A and BCL-2 in A549-generated xenografts by immunohistochemistry (upper panels) and TUNEL assay (lower panel). **d** Quantification analysis of the staining intensity and **e** the apoptotic rate. **f** and **g** MiR-130b mimic decreased the level of PPARγ in A549-generated xenografts, but increased VEGF-A and BCL-2. Scale bar, 50 μm. CTRL: control; TUNEL, terminal deoxynucleotidyl transferase-mediated uridine 5’-triphosphate-biotin nick end labeling. Each bar represents the mean ± SD. Results are representative of three independent experiments. *p < 0.05, #*p* < 0.001

## Discussion

The present study indicates that miR-130b increases the expression of VEGF-A and BCL-2 but suppresses PPARγ and apoptosis. Importantly, we demonstrate that VEGF-A targets BCL-2 and promotes the aggressiveness of lung cancer cells via BCL-2-mediated suppression of apoptosis. These data highlight the critical role of miR-130b in promoting lung cancer progression through PPARγ/VEGF-A/BCL-2-mediated suppression of apoptosis (Fig. 8). Another major finding of this study is that PPARγ antagonist GW9662 attenuates the effect of miR-130b inhibition on VEGF-A/BCL-2-mediated apoptosis and downstream gene expressions. Furthermore, immunoprecipitation demonstrates the interaction between PPARγ and VEGF-A, supporting the notion that miR-130b plays a critical role in regulating lung cancer cell aggressiveness and apoptosis through the PPARγ/VEGF-A axis. However, neither PPARγ nor VEGF-A siRNAs had feedback regulatory effects on the miR-130b expression. This suggests that miR-130b acts as the upstream of the PPARγ/VEGF-A axis in mediating apoptosis and downstream gene expressions.

**Fig. 8:** Schematic diagram of microRNA-130b in promoting lung cancer progression via PPARγ/VEGF-A/BCL-2-mediated suppression of apoptosis

Studies have demonstrated that miR-130b suppresses migration and invasion of colorectal cancer cells through downregulation of Integrin-β1 [24]. MiR-130b may promote hepatocellular carcinoma cell migration and invasion by inhibiting PPARγ and subsequently inducing EMT [18, 25]. MiR-130b also plays an important profibrotic role in skin fibrosis and enhances TGF-β signaling through repression of PPARγ [26]. Moreover, varied expression levels of miR-130b have been found in endometrial [27], gastric [28] and bladder [29] cancer regulating different signaling molecules. We found that miR-130b, by targeting PPARγ, promotes aggressiveness through VEGF-A-mediated suppression of apoptosis in lung cancer. These studies demonstrate that miR-130b plays a role in regulating tumor progression.

Functionally, our data indicate that miR-130b not only exhibits a potent oncogenic role, in agreement with other recent reports [30], but also suppresses lung cancer cell apoptosis through VEGF-A-mediated up-regulation of BCL-2, the classical anti-apoptotic gene. In addition, knocking down VEGF-A caused a significant reduction in BCL-2 protein level and decreased luciferase activity. These results together suggest that VEGF-A interacts with BCL-2 in mediating lung cancer cell apoptosis. It has been demonstrated that in wild-type p53 expressing cells, miR-130b directly represses Zinc finger E-box-binding homeobox 1 (ZEB1), opposing EMT and invasive phenotypes. However, in the context of gain-of-function p53 mutations, mutant p53 triggers EMT by indirectly inducing ZEB1 expression through negative regulation of miR-130b [27]. Undoubtedly, miR-130b exerts a critical function in regulating cell apoptotic processes. Our results have revealed for the first time that miR-130b, through up-regulating the BCL-2 signaling, enhances lung cancer progression and inhibits cell apoptosis. Future studies exploring the significance of circulating miR-130b in lung cancer development and progression may provide possible evidences for early detection and screening of lung cancer risk factors. Our results have shown that miR-130b promotes lung cancer progression through PPARγ/VEGF-A/BCL-2-mediated suppression of apoptosis.

Lines of evidence have demonstrated the link between miRNA dysregulation with malignant transformation in a variety of cancers [31–33]. Previous report [34] and our present results identify miR-130b as an important signature in lung cancer. MiR-130b up-regulation has been detected in lung adenocarcinoma and squamous cell carcinoma and confers advanced tumor stage, poor differentiation and unfavorable prognosis of lung cancer patients. This is in line with other studies showing that miR-130b up-regulation correlates with the clinical stage of gastric [35] and esophageal carcinoma [30]. However, we found that in lung cancer tissues, cases with high miR-130b expression level did not correlate positively with lymph node metastases and larger tumor size. We assume that factors, like the tumor microenvironment or other growth factors, also contributed to the lymph node metastasis and growth of lung tumors. In addition, this could also be in part due to the limited sample size analyzed in the present study, which needs further investigations in expanded samples.

## Conclusions

We demonstrate that miR-130b targets PPARγ and suppresses lung cancer cell apoptosis through the VEGF-A/BCL-2 pathway. High miR-130b expression confers unfavorable prognosis of lung cancer patients. These findings indicate clinical values of our study and that miR-130b is a potential new therapeutic target for lung cancer diagnosis and treatment.

## Abbreviations

AD, adenocarcinoma; anti-M, anti-miR-130b; anti-MC, anti-miR-130b control; EMT, epithelial to mesenchymal transition; miR-130b, microRNA-130b; NL, normal lung; NSCLC, non-small-cell lung cancer; NT siRNA, non-targeting small interference RNA; PPARγ, peroxisome proliferator-activated receptor γ; PPRE, PPAR-response element; SD, standard deviation; SQ, squamous cell carcinoma; TUNEL, terminal deoxynucleotidyl transferase-mediated uridine 5’-triphosphate-biotin nick end labeling; VEGF-A, vascular endothelial growth factor-A; ZEB1, zinc finger E-box-binding homeobox 1

## Additional file

Additional file 1: MiR-130b mimic enhances lung cancer cell aggressiveness via PPARγ/VEGF-A/BCL-2-mediated suppression of apoptosis. (A) Representative images of A549 cells treated with miR-130b mimic and co-labeled for PPARγ (green) and VEGF-A (red) (scale bar, 50 μm). (B) Representative images of A549 cells treated with miR-130b mimic and labeled for BCL-2 (green) (scale bar, 50 μm). (C and D) MiR-130b mimic decreased PPARγ, but increased VEGF-A and BCL-2. (E) MiR-130b mimic caused a significant decrease in the luciferase activity of wt 3'-UTR of *PPARγ*. (F) A faster proliferation rate in cells treated with miR-130b mimic compared with controls. (G) Increased number of invaded cells with miR-130b mimic treatment (scale bar, 100 μm). (H) Longer migrated distance in cells treated with miR-130b mimic at indicated time points. (I) Increased colonies in cells treated with miR-130b mimic at 48 hours time point. (J) Decreased apoptotic cells treated with miR-130b mimic compared with controls. (K) Decreased apoptotic rate in cells treated with miR-130b mimic (scale bar, 50 μm). NC: normal control; miR-NC: miR-130b control; miR-130bm: miR-130b mimic; TUNEL, terminal deoxynucleotidyl transferase-mediated uridine 5’-triphosphate-biotin nick end labeling. Each bar represents the mean ± SD. Results are representative of three independent experiments. *p < 0.05, #p < 0.001. (DOC 2779 kb)
